# Cardiogenic Shock With Reverse Takotsubo Pattern Secondary to Pheochromocytoma: A Case Report

**DOI:** 10.7759/cureus.19600

**Published:** 2021-11-15

**Authors:** Angkawipa Trongtorsak, Natapat Chaisidhivej, Jakrin Kewcharoen, Poranee Ganokroj, Artit Torpongpun

**Affiliations:** 1 Internal Medicine, AMITA Health Saint Francis Hospital, Evanston, USA; 2 Department of Medicine, Einstein Medical Center Philadelphia, Philadelphia, USA; 3 Division of Cardiovascular Medicine, Loma Linda University Health, Loma Linda, USA; 4 Division of Endocrinology and Metabolism, Department of Medicine, Faculty of Medicine, Chulalongkorn University, Bangkok, THA; 5 Division of Cardiovascular Medicine, Department of Medicine, Chonburi Hospital, Chonburi, THA

**Keywords:** cariogenic shock, pheochromocytoma, cardiomyopathy, reverse takotsubo cardiomyopathy, catecholamine cardiomyopathy

## Abstract

Pheochromocytoma is a rare catecholamine-secreting neuroendocrine tumor arising from chromaffin cells. Acute catecholamine-mediated cardiomyopathy secondary to pheochromocytoma is rare, but life-threatening. We report a case of a 50-year-old man who presented with chest pain with electrocardiography showing ST elevation in V2-4. He was transferred to cardiac catheterization laboratory for coronary angiography immediately. However, the results showed no evidence of coronary artery occlusions and the left ventriculography revealed hypokinesia of basal part with poor left ventricular ejection fraction. Further investigation confirmed pheochromocytoma-related reversible cardiomyopathy.

## Introduction

Pheochromocytoma is a rare neuroendocrine tumor that arises from chromaffin cells. The common presentations are headache, sweating, palpitations and paroxysmal hypertension. Cardiac manifestations of pheochromocytoma include arrhythmias, myocardial ischemia, reversible cardiomyopathy and even cardiogenic shock. Patients with pheochromocytoma can present with reverse Takotsubo-like cardiomyopathy. It is defined as a reversible cardiomyopathy with hypokinesia at the basal wall of the heart [1-3].

## Case presentation

A 50-year-old Asian man with past medical history of hypertension presented to the emergency department with a dull chest pain associated with severe dyspnea, nausea, and vomiting. His blood pressure was 199/90 mmHg, heart rate was 120 beats/minute, respiratory rate was 30 breaths/minute and body temperature was 37.7 degrees Celsius. During the initial evaluation, his blood pressure suddenly dropped to 86/58 mmHg. His 12-lead electrocardiogram (ECG) showed ST elevation at V2-4 and inverted T wave at V1 (Figure 1). His chest x-ray showed moderate pulmonary edema (Figure 2). He was diagnosed with ST-elevation myocardial infarction (STEMI) with cardiogenic shock leading to acute decompensated heart failure. He was intubated and underwent emergent cardiac catheterization. The cardiac catheterization revealed no coronary artery occlusion, but the left ventriculography showed poor left ventricular ejection fraction (LVEF) with basal hypokinesia and preserved apical wall motion (Figure 3). Transthoracic echocardiogram was performed five days after the admission and LVEF had improved to 73% with normal size chambers. Reverse Takotsubo cardiomyopathy was suspected.

**Figure 1:** The patient’s admission ECG shows ST elevation at V2-4 and inverted T at V1

**Figure 2:** The patient’s chest x-ray shows moderate pulmonary edema

**Figure 3:** Left ventriculogram shows hypokinesia of basal segment and excessive apical motion. A: Diastolic phase, B: Systolic phase

Patient was diagnosed with essential hypertension since he was 35 years old. For the past year, he had been experiencing several episodes of chest pain at rest, palpitation, sweating and headache. He was referred to a cardiologist for an exercise stress test and coronary angiography (CAG) which results came back as negative. He had been treated as stable coronary for a few months and recently received atenolol one week before the admission. The patient denied any emotional or physical stressors.

Further investigations showed a high level of urinary vanillylmandelic acid (VMA) with a normal level of plasma aldosterone concentration, plasma renin activity and serum cortisol (Table 1). Computed tomography (CT) scan of adrenal glands showed a 5.7x6.3x6.7 cm^3^ right adrenal mass (Figure 4). Pheochromocytoma-related cardiomyopathy was suspected. After receiving adequate medical control, the patient underwent an uncomplicated right adrenalectomy and the pathological report confirmed the diagnosis of pheochromocytoma (Figures 5, 6).

**Table 1:** Laboratory findings TSH: thyroid-stimulating hormone, FT3: free triiodothyroinine, FT4: free thyroxine, PRA: plasma renin activity, VMA: vanillylmandelic acid

Parameter	Patient value	Normal range
Serum		
Cortisol	13.7	AM 6.2-19.4, PM 2.3-11.9 mcg/dl
TSH	3.7	0.27-4.2 uIU/ml
FT3	2.5	2-4.4 pg/ml
FT4	1.43	0.93-1.7 ng/dl
Aldosterone	7	supine 1-16, upright 4-31 ng/dl
PRA	8.21	supine 0.2-1.6 upright 0.5-4 ng/ml/hour
Urine		
Metanephrine	9,624	< 1,777 nmol/day
Normetanephrine	49,213	<3,279 nmol/day
VMA	29	1-11 mg/day

**Figure 4:** CT scan shows right adrenal mass (Left: circle, Right: arrowhead)

**Figure 5:** Right adrenal gland sized 6.8x6.7x5.5 cm with hemorrhagic area

**Figure 6:** Microscopic appearance of adrenal tumor A: Normal adrenal cortex and tumor in adrenal medulla B,C,D: The tumor consists of spindle cells with round nuclei and prominent nucleolus arranged in small nests (zellballen) separated by rich vascular network

## Discussion

Pheochromocytoma can arise from either adrenal medulla (80-85%) or extra-adrenal paraganglia. The prevalence of pheochromocytoma was reported to be 0.1-0.4% in patients with hypertension [1]. Clinical presentations of pheochromocytoma can vary, but the common clinical signs and symptoms include hypertension, headache, sweating, tachycardia and anxiety [1]. Hypertension found with pheochromocytoma is usually paroxysmal; however, some patients may have sustained hypertension [1-3]. Pheochromocytoma occurs either hereditary or sporadic. Hereditary pheochromocytoma can be found in neurofibromatosis type 1, multiple endocrine neoplasia type2 (MEN 2A, MEN 2B), von Hippel-Lindau syndrome and the familial paragangliomas [4].

The diagnosis of pheochromocytoma is often challenging due to the many different clinical presentations. All patients who are suspected for pheochromocytoma should undergo biochemical testing for catecholamine excess. Biochemical tests include a measurement of plasma catecholamines, urinary metanephrine and normetanephrine and urinary vanillylmandelic acid (VMA) [5-7]. After biochemical testing results as positive, further imaging study should be performed to localize the tumor. CT scan of the whole abdomen is the most often used imaging test for an initial localization of the tumor due to the cost-effectiveness and high sensitivity [7].

Currently, the treatment of choice is surgical resection of the tumor. However, adequate preoperative management is required to prevent a catecholamine-induced hypertensive crisis. Blood pressure control can be achieved by using an a-blocker and/or b-blocker. Phenoxybenzamine, a non-selective a-blocker, is recommended for 10-14 days to control blood pressure and prevent a hypertensive crisis [5]. A b-blocker is often required when patients develop tachycardia or arrhythmia but it should never be used before an a-blocker because patients can develop hypertensive crisis due to an unopposed a-adrenergic receptor stimulation [4].

Acute catecholamine-mediated cardiomyopathy associated pheochromocytoma is rare but life-threatening. It has been reported that patients can present with transient reversible cardiomyopathy in Takotsubo or diffuse hypokinesia pattern [8]. Similar to our case, Tagawa et al. reported a case of a young lady who presented with reverse Takotsubo cardiomyopathy and ventricular arrhythmia secondary to pheochromocytoma [9]. However, it was her first presentation at that time. Examining these studies, the decreased LVEF usually resolves within a few days. The cardiac manifestation is believed to be caused by a massive release of catecholamine. The mechanism of cardiac muscle injury from catecholamine is still unclear; however, it is hypothesized that the sympathetic hyperactivity can cause a direct toxic effect on the cardiac muscle, increase in oxygen demand with a decrease in oxygen supply and induce coronary vasoconstriction [10-11]. The variation of hypokinetic area may be due to an asymmetric distribution of adrenergic receptors [12]. Compared to the usual Takotsubo pattern, reverse Takotsubo tends to present in the younger age. The mean age of patients with Takotsubo and reverse Takotsubo are 62 and 36 years old respectively [13]. The presentation of the reverse Takotsubo cardiomyopathy in the younger patients may be due to the large number of adrenergic receptors in the basal area [13]. According to other reports which patients usually presented with acute severe symptoms, this patient had developed chronic atypical chest pain with normal coronary angiogram before presenting with sudden severe chest pain with cardiogenic shock. However, the role of coronary angiography and echocardiography (or ventriculography) are prerequisites for diagnostic confirmation of reverse Takotsubo cardiomyopathy. For the precipitating cause in this patient, atenolol seemed to be the only reason since he was healthy, his medical condition was quite controlled and had no emotional or physical stress [8-9].

Apart from emotional or physical distress, pheochromocytoma and other secondary causes should be suspected in patients presenting with Takotsubo or reverse Takotsubo cardiomyopathy. Moreover, patients with angina pain with no significant coronary artery stenosis on CAG can be due to secondary causes such as pheochromocytoma.

## Conclusions

The cardiac manifestations are not common but are documented as patients may present with arrhythmia, chest pain or reversible catecholamine cardiomyopathy. The treatment of choice is surgical resection. Before an operation, proper perioperative management is required in order to prevent a catecholamine-induced hypertensive crisis. A b-blocker should never be used before an a-blocker because it can induce hypertensive crisis due to unopposed a-adrenergic receptors.
